The article "Systematic Identification of lncRNA-Associated ceRNA Networks in Immune Thrombocytopenia" was published in 2020. Journal: Comput Math Methods Med.

# Systematic Identification of lncRNA-Associated ceRNA Networks in Immune Thrombocytopenia

**DOI:** 10.1155/2020/6193593

**Published:** 2020-06-30

**Authors:** Zhenwei Fan, Xuan Wang, Peng Li, Chunli Mei, Min Zhang, Chunshan Zhao, Yan Song

**Affiliations:** ^1^Nursing College of Beihua University, Jilin 132013, China; ^2^Department of Hematology, Affiliated Hospital of Beihua University, Jilin 132013, China; ^3^Department of Oncology, Jilin Central Hospital, Jilin 132000, China

## Abstract

Primary immune thrombocytopenia (ITP) is an autoimmune disease. However, the molecular mechanisms underlying ITP remained to be further investigated. In the present study, we analyzed a series of public datasets (including GSE43177 and GSE43178) and identified 468 upregulated mRNAs, 272 downregulated mRNAs, 134 upregulated lncRNAs, 23 downregulated lncRNAs, 29 upregulated miRNAs, and 39 downregulated miRNAs in ITP patients. Then, we constructed protein-protein interaction networks, miRNA-mRNA and lncRNA coexpression networks in ITP. Bioinformatics analysis showed these genes regulated multiple biological processes in ITP, such as mRNA nonsense-mediated decay, translation, cell-cell adhesion, proteasome-mediated ubiquitin, and mRNA splicing. We thought the present study could broaden our insights into the mechanism underlying the progression of ITP and provide a potential biomarker for the prognosis of ITP.

## 1. Introduction

Primary immune thrombocytopenia (ITP) is an autoimmune disease characterized by a decrease in platelets due to platelet destruction and insufficient platelet production [1, 2]. Previous studies had showed the increasing antiplatelet antibodies produced by B cells, and the aberrant functions of T lymphocytes were involved in regulating the progression of ITP [3]. However, the mechanisms regulating ITP progression remained to be further investigated.

In the past decades, increasing evidence showed more than 90% human genome could not be translated to proteins. Noncoding RNAs, such as miRNAs and lncRNAs, played important roles in the progression of human diseases [4]. miRNAs were a type of ncRNAs with 19-25 bps in length and regulated gene expression and protein translation by targeting 3-UTR of mRNAs. Previous studies showed miRNAs were dysregulated and associated with the regulation of ITP. For example, miR-99a expression was overexpressed in CD4+ cells [5], while expression of miR-182-5p and miR-183-5p was overexpressed in ITP. MIR130A was downregulated and suppressed TGFB1 and IL18 in ITP [6]. Meanwhile, MIR409-3p was also reported to be reduced in ITP samples [7]. Long noncoding RNAs (lncRNAs) are a class of ncRNAs longer than 200 nucleotides with no protein-coding potential. The roles of lncRNAs in autoimmune diseases were also implicated. Wang et al. found that lncRNA TMEVPG1 expression was lower than that in healthy control samples [8]. Liu et al. identified a total of 1177 and 632 lncRNAs were significantly upregulated or downregulated in ITP patients compared to normal samples [9].

The article "Systematic Identification of lncRNA-Associated ceRNA Networks in Immune Thrombocytopenia" was published in 2020. Journal: Comput Math Methods Med.

In the present study, we screened differently expressed mRNAs, miRNAs, and lncRNAs in ITP compared to normal samples using two public datasets, GSE43177 and GSE43178. Then, bioinformatics analysis was employed to predict the potential functions of differently expressed mRNAs, miRNAs, and lncRNAs in ITP. This study could provide useful information for exploring therapeutic candidate targets and new molecular biomarkers for ITP.

## 2. Material and Methods

### 2.1. Microarray Data and Data Preprocessing

Gene expression datasets were obtained from the NCBI Gene Expression Omnibus (GEO) (http://www.ncbi.nlm.nih.gov/geo) with accession numbers GSE43177 [10] and GSE43178 [10]. The 10 normal and 9 ITP samples were included in the GSE43177 dataset. Meanwhile, the 9 normal and 9 ITP samples were included in GSE43178 dataset.

### 2.2. lncRNA Classification Pipeline

In order to evaluate the expression of lncRNAs in microarray data, a pipeline was employed to identify the probe sets uniquely mapped to lncRNAs from the Affymetrix array. A total of 2448 annotated lncRNA transcripts with corresponding Affymetrix probe IDs were obtained. The cutoff values used for selecting differentially expressed lncRNAs were fold change ≥ 2 and *P* < 0.05.

### 2.3. Prediction of the Targets of miRNAs

To obtain valuable insights into the potential mechanisms of miRNAs, a bioinformatics analysis was performed to identify the target genes of miRNAs using starBase. starBase is a database that combines data from six prediction programs: TargetScan, PicTar (http://www.pictar.org/), miRanda (http://www.microrna.org/microrna/home.do), PITA (http://www.genie.weizmann.ac.il/index.html), RNA22 (http://www.cm.jefferson.edu/rna22/), and CLIP-Seq (http://www.starbase.sysu.edu.cn/).

### 2.4. Functional Group Analysis

GO analysis and KEGG analysis were employed to determine the biological functions of the identified differentially expressed mRNAs, based on the freely available online MAS 3.0 system from CapitalBio Corporation (http://bioinfo.capitalbio.com/mas3/; Beijing, China). The *P* value (hypergeometric *P* value) denotes the significance of the pathway associated with the conditions. *P* < 0.05 was considered to indicate a statistically significant difference.

### 2.5. Protein-Protein Interaction Network Mapping

We followed the methods of Chen et al. [11]. The Search Tool for the Retrieval of Interacting Genes/Proteins (STRING) [12] online software (https://string-db.org) was utilized to assess the potential interactions. The interactions of the proteins encoded by the differently expressed genes were searched using STRING online software, and the combined score of >0.4 was used as the cutoff criterion. Cytoscape software (http://www.cytoscape.org) was used for the visualization of the PPI network.

The article "Systematic Identification of lncRNA-Associated ceRNA Networks in Immune Thrombocytopenia" was published in 2020. Journal: Comput Math Methods Med.

### 2.6. Construction of the Coexpression Network between Differentially Expressed mRNAs and lncRNAs

The Pearson correlation coefficient of DEG-lncRNA pairs was calculated according to their expression values. The coexpressed DEG-lncRNA pairs with an absolute value of the Pearson correlation coefficient of ≥0.8 were selected, and the coexpression network was visualized by using Cytoscape software.

## 3. Result

### 3.1. Identification of Differently Expressed mRNAs, lncRNAs, and miRNAs in Immune Thrombocytopenia

First, we analyzed a public dataset GSE43177 to identify differently expressed mRNAs in ITP samples compared to healthy control samples. Subsequently, differential expression analysis was conducted by using GEO2R (∣log2FC | >1 and adj. *P* value < 0.05). A total 740 genes were identified as DEGs in ITP, including 468 upregulated genes and 272 downregulated genes. These upregulated and downregulated significant DEGs were present using hierarchical clustering (Figure 1(a)).

By reannotating the gene probes in GSE43177, we found that 1561 lncRNA probes were included in this dataset. Among them, 157 lncRNAs were found to be dysregulated in ITP. 134 lncRNAs were overexpressed and 23 lncRNAs were downregulated in ITP samples compared to healthy control samples (Figure 1(b)).

Then, we analyzed a public dataset GSE43178 to identify differently expressed miRNAs in ITP. 68 miRNAs were observed to be differentially expressed, including 29 upregulated miRNAs and 39 downregulated miRNAs. The heat map of DEGs in the ITP and control stromal cells is shown in Figure 1(c).

### 3.2. Construction of the PPI Network Mediated by DEGs in ITP

Subsequently, the PPI network analyses were conducted to reveal the relationships among DEGs. As shown in Figure 2, a total of 404 nodes and 1391 interactions were identified in this PPI network. Interestingly, three sub-PPI networks (red network, green network, and purple network) were identified. The red network included 24 nodes and 132 edges. The green network included 11 nodes and 55 edges. And the purple network included 8 nodes and 28 edges. Seven DEGs played a more important regulatory role in this network by connecting with more than 10 different DEGs, including MMP9, LCN2, DYNLL2, CKAP4, FOLR3, FBXO32, and PLD1.

The article "Systematic Identification of lncRNA-Associated ceRNA Networks in Immune Thrombocytopenia" was published in 2020. Journal: Comput Math Methods Med.

### 3.3. Construction of miRNA-DEG Networks in ITP

Furthermore, we used TargetScan and starBase [13] to predict the downstream targets of differently expressed miRNAs in ITP. Then, a miRNA-DEG network was constructed using Cytoscape software (Figure 3). A total of 26 miRNAs and 279 mRNAs were included in this network. Interestingly, we found that hsa-miR-30a, hsa-let-7b, hsa-miR-30e, hsa-miR-200a, hsa-miR-520e, hsa-miR-494, hsa-miR-543, hsa-miR-302d, hsa-miR-377, hsa-miR-363, and hsa-miR-200b played crucial roles in ITP.

### 3.4. Construction of lncRNA-mRNA Coexpression Networks in ITP

In order to reveal the potential functions of lncRNAs in ITP, we first conducted lncRNA coexpression analysis based on their expression levels in ITP samples. Then, the lncRNA-mRNA pairs with the value of the absolute Pearson correlation coefficient ≥ 0.75 were selected for network construction. The lncRNA coexpression networks in ITP were constructed using Cytoscape 3.0 [14] (http://www.cytoscape.org/).

As presented in Figure 4, 136 lncRNAs, 430 mRNAs, and 1415 edges were contained in this coexpression network. Based on the coexpression network analysis, 8 lncRNAs (LOC101927237, LINC00515, LOC101927066, LOC440028, RP11-161D15.1, LOC101929312, AX747630, and LOC100506406) were identified as key regulators in ITP and regulated more than 55 dysregulated mRNAs in ITP (Figure 3).

### 3.5. Bioinformatics Analysis of mRNAs, miRNAs, and lncRNAs in ITP

In Figure 5, bioinformatics analysis showed DEGs in ITP were associated with the mRNA nonsense-mediated decay, translation, cell-cell adhesion, proteasome-mediated ubiquitin, and mRNA splicing, via spliceosome, protein polyubiquitination, viral process, autophagy, rRNA processing, and macroautophagy. ITP-related miRNAs were involved in regulating the cytoskeleton-dependent intracellular transport, negative regulation of epithelial cell proliferation, protein localization, proteasome, nuclear DNA replication, nucleotide excision repair, branched-chain amino acid catabolic process, regulation of mitophagy, cellular response to cAMP, and negative regulation of transcription. ITP-related lncRNAs were involved in regulating the positive regulation of inflammatory response, cellular response to cGMP, ephrin receptor signaling pathway, chronic inflammatory response, forelimb morphogenesis, stem cell population maintenance, cell junction assembly, positive regulation of cell growth, chemical synaptic transmission, and inflammatory response.

Bioinformatics analysis showed DEGs in ITP were associated with the oxytocin signaling pathway, glutamatergic synapse, choline metabolism in cancer, dopaminergic synapse, FoxO signaling pathway, hypertrophic cardiomyopathy (HCM), ovarian steroidogenesis, thyroid hormone synthesis, serotonergic synapse, and metabolic pathways. ITP-related miRNAs were associated with endocytosis, pyrimidine metabolism, prostate cancer, drug metabolism-other enzymes, FoxO signaling pathway, glioma, choline metabolism in cancer, thyroid hormone synthesis, hepatitis B, and metabolic pathways. ITP-related lncRNAs were associated with glutamatergic synapse, endocytosis, serotonergic synapse, dopaminergic synapse, arrhythmogenic right ventricular cardiomyopathy, platelet activation, estrogen signaling pathway, thyroid hormone synthesis, FoxO signaling pathway, and focal adhesion.

The article "Systematic Identification of lncRNA-Associated ceRNA Networks in Immune Thrombocytopenia" was published in 2020. Journal: Comput Math Methods Med.

## 4. Discussion

ITP is an autoimmune disorder. The increasing antiplatelet antibodies produced by B cells, and the aberrant functions of T lymphocytes were involved in regulating the ITP. Previous studies revealed that the dysregulation of multiple genes, such as miRNAs and lncRNAs, contributed to the progression of ITP. For example, MIR130A, MIR409-3p, and lncRNA TMEVPG1 were downregulated in ITP. Moreover, Qian et al. identified a total of 1809 lncRNAs were significantly dysregulated in ITP patients compared to normal samples. Better understanding of the regulation of ITP is very crucial for the discovery of therapeutic targets for the treatment of this disease.

The present study screened differently expressed mRNAs, lncRNAs, and miRNAs in ITP. A total 740 genes were identified as DEGs in ITP, including 468 upregulated genes and 272 downregulated genes. Subsequently, a PPI network, including 404 nodes and 1391 interaction, was constructed to identify hub regulators in ITP. Seven DEGs played a more important regulatory role in this network by connecting with more than 10 different DEGs, including MMP9, LCN2, DYNLL2, CKAP4, FOLR3, FBXO32, and PLD1. This is the first time their regulatory roles in ITP were revealed. Notably, PLD1 had been demonstrated to play an important role in autoimmune diseases. PLD1 mediated lymphocyte adhesion and migration in autoimmune encephalomyelitis [15]. PLD1 regulated the expression of proinflammatory genes in rheumatoid arthritis synovial fibroblasts [16]. Bioinformatics analysis showed DEGs in ITP were associated with the mRNA nonsense-mediated decay, translation, cell-cell adhesion, proteasome-mediated ubiquitin, and mRNA splicing, via spliceosome, protein polyubiquitination, viral process, autophagy, rRNA processing, and macroautophagy.

Increasing evidence indicated that miRNAs and lncRNAs are essential in regulating gene expression, cell proliferation, apoptosis, and migration. However, the detail functions and special expression pattern of miRNAs and lncRNAs in ITP remained largely unclear. Meanwhile, we identified 134 upregulated lncRNAs, 23 downregulated lncRNAs, 29 upregulated miRNAs, and 39 downregulated miRNAs in ITP patients. Furthermore, we constructed the miRNA-DEG network and lncRNA coexpression network to explore their functions in ITP. Interestingly, 8 lncRNAs (LOC101927237, LINC00515, LOC101927066, LOC440028, RP11-161D15.1, LOC101929312, AX747630, and LOC100506406) were identified as key regulators in ITP. Among them, LINC00515 was reported to promote multiple myeloma autophagy and chemoresistance though the miR-140-5p/ATG14 axis [17]. However, the functions of most lncRNAs were unknown in human diseases. Bioinformatics analysis showed ITP-related lncRNAs were involved in regulating the positive regulation of inflammatory response, cellular response to cGMP, ephrin receptor signaling pathway, chronic inflammatory response, forelimb morphogenesis, stem cell population maintenance, cell junction assembly, positive regulation of cell growth, chemical synaptic transmission, and inflammatory response.

The article "Systematic Identification of lncRNA-Associated ceRNA Networks in Immune Thrombocytopenia" was published in 2020. Journal: Comput Math Methods Med.

Several limitations should be noted in this study. First, this study was mainly based on bioinformatics analysis. Therefore, the functional validation should be conducted in the near future. Second, the sample size in this study was small. We should collect more clinical samples to detect the expression of the key mRNAs, miRNAs, and lncRNAs in the progression of ITP.

In conclusion, our integrative analysis identified key mRNAs, miRNAs, and lncRNAs in the progression of ITP. Bioinformatics analysis showed these genes regulated multiple biological processes in ITP, such as mRNA nonsense-mediated decay, translation, cell-cell adhesion, proteasome-mediated ubiquitin, and mRNA splicing. We thought the present study could broaden our insights into the mechanism underlying the progression of ITP and provide a potential biomarker for the prognosis of ITP.

## Figures and Tables

**Figure 1:** Heat map of differently expressed mRNAs, lncRNAs, and miRNAs in immune thrombocytopenia. Heat map depicts different expression of (a) mRNAs, (b) lncRNAs, and (c) miRNAs in immune thrombocytopenia. Shades of yellow and deongaree represent log2 gene expression values.

**Figure 2:** PPI network of differently expressed mRNAs in ITP. The PPI network consists of 404 mRNAs. The red subnetwork included 24 nodes and 132 edges. The green subnetwork included 11 nodes and 55 edges. And the purple subnetwork included 8 nodes and 28 edges.

**Figure 3:** PPI network of differently expressed mRNA-target miRNA in ITP. The PPI network consists of 26 miRNAs and correlated 279 target mRNAs. The lilac dot represents mRNA; the green dot represents miRNA.

The article "Systematic Identification of lncRNA-Associated ceRNA Networks in Immune Thrombocytopenia" was published in 2020. Journal: Comput Math Methods Med.

**Figure 4:** Coexpression networks of lncRNAs in ITP. The coexpression network consists of 136 lncRNAs and correlated 430 mRNAs. The blue dot represents mRNA; the green dot represents lncRNA.

**Figure 5:** GO analysis and KEGG analysis of mRNAs, miRNAs, and lncRNAs in ITP. (a) Biological process analysis of the related mRNAs. (b) KEGG pathway analysis of the related mRNAs. (c) Biological process analysis of the related miRNAs. (d) KEGG pathway analysis of the related miRNAs. (e) Biological process analysis of the related lncRNAs. (f) KEGG pathway analysis of the related lncRNAs.

## Data Availability

Gene expression datasets were obtained from the NCBI Gene Expression Omnibus (GEO) (http://www.ncbi.nlm.nih.gov/geo) with accession numbers GSE43177 and GSE43178.

## Abbreviations

ITP: Immune thrombocytopenia
lncRNAs: Long noncoding RNAs
STRING: Search Tool for the Retrieval of Interacting Genes/Proteins
GEO: Gene Expression Omnibus.

## References

[1] Barsam S. J., Psaila B., Forestier M. (2011). Platelet production and platelet destruction: assessing mechanisms of treatment effect in immune thrombocytopenia. *Blood*.

[2] Yazdanbakhsh K., Zhong H., Bao W. (2013). Immune dysregulation in immune thrombocytopenia. *Seminars in Hematology*.

[3] Chistiakov D. A. (2005). Immunogenetics of Hashimoto's thyroiditis. *Journal of Autoimmune Diseases*.

[4] Esteller M. (2011). Non-coding RNAs in human disease. *Nature Reviews Genetics*.

[5] Warth S. C., Hoefig K. P., Hiekel A. (2015). Induced miR-99a expression represses Mtor cooperatively with miR-150 to promote regulatory T-cell differentiation. *The EMBO Journal*.

[6] Zhao H., Li H., du W. (2014). Reduced *MIR130A* is involved in primary immune thrombocytopenia via targeting *TGFB1* and *IL18*. *British Journal of Haematology*.

[7] Chang M., Nakagawa P. A., Williams S. A. (2003). Immune thrombocytopenic purpura (ITP) plasma and purified ITP monoclonal autoantibodies inhibit megakaryocytopoiesis in vitro. *Blood*.

[8] Wang J., Peng H., Tian J. (2016). Upregulation of long noncoding RNA TMEVPG1 enhances T helper type 1 cell response in patients with Sjögren syndrome. *Immunologic Research*.

[9] Liu W. J., Bai J., Guo Q. L., Huang Z., Yang H., Bai Y. Q. (2016). Role of platelet function and platelet membrane glycoproteins in children with primary immune thrombocytopenia. *Molecular Medicine Reports*.

[10] Jernås M., Nookaew I., Wadenvik H., Olsson B. (2013). MicroRNA regulate immunological pathways in T-cells in immune thrombocytopenia (ITP). *Blood*.

[11] Chen L., Zhang Y., Rao Z., Zhang J., Sun Y. (2018). Integrated analysis of key mRNAs and lncRNAs in osteoarthritis. *Experimental and Therapeutic Medicine*.

The article "Systematic Identification of lncRNA-Associated ceRNA Networks in Immune Thrombocytopenia" was published in 2020. Journal: Comput Math Methods Med.

[12] Szklarczyk D., Gable A. L., Lyon D. (2019). STRING v11: protein–protein association networks with increased coverage, supporting functional discovery in genome-wide experimental datasets. *Nucleic Acids Research*.

[13] Yang J. H., Li J. H., Shao P., Zhou H., Chen Y. Q., Qu L. H. (2011). starBase: a database for exploring microRNA–mRNA interaction maps from Argonaute CLIP-Seq and Degradome-Seq data. *Nucleic Acids Research*.

[14] Shannon P., Markiel A., Ozier O. (2003). Cytoscape: a software environment for integrated models of biomolecular interaction networks. *Genome Research*.

[15] Frohman M. A. (2015). The phospholipase D superfamily as therapeutic targets. *Trends in Pharmacological Sciences*.

[16] Müller-Ladner U., Kriegsmann J., Franklin B. N. (1996). Synovial fibroblasts of patients with rheumatoid arthritis attach to and invade normal human cartilage when engrafted into SCID mice. *American Journal of Pathology*.

[17] Meng Y., Gao R., Ma J. (2017). MicroRNA-140-5p regulates osteosarcoma chemoresistance by targeting HMGN5 and autophagy. *Scientific Reports*.

